# Urine cell‐free DNA as a promising biomarker for early detection of non‐small cell lung cancer

**DOI:** 10.1002/jcla.23321

**Published:** 2020-04-13

**Authors:** Sai Ren, Xiao-Dong Ren, Li-Fang Guo, Xue-Mei Qu, Mei-Yun Shang, Xiao-Tian Dai, Qing Huang

**Affiliations:** ^1^ Department of Laboratory Medicine Daping Hospital Army Medical University Chongqing China; ^2^ Department of Pulmonology Southwest Hospital Army Medical University Chongqing China

**Keywords:** DNA integrity, LINE1 repeat sequences, non‐small‐cell lung cancer, quantitative real‐time PCR, urine cell‐free DNA

## Abstract

**Background:**

While blood‐derived cell‐free DNA has been shown to be a candidate biomarker able to provide diagnostic and prognostic insight in cancer patients, little is known regarding the potential application of urine cell‐free DNA (ucfDNA) in diagnosis of cancer. Thus, the aim of this study was to investigate ucfDNA concentration and integrity index as potential biomarkers for early detection of non‐small‐cell lung cancer (NSCLC).

**Methods:**

Urine samples were collected from 35 healthy controls and 55 NSCLC patients at various tumor node metastasis (TNM) stages. Two long interspersed nuclear element 1 (LINE1) fragments (LINE1‐97 and 266 bp) were quantified via quantitative real‐time PCR (qPCR). DNA integrity index was calculated as the ratio of LINE1‐266/LINE‐97.

**Results:**

LINE1 fragments concentrations of ucfDNA (LINE1‐97, 266 bp) were significantly higher in NSCLC patients with stage III/IV than in stage I/II and in healthy controls. The receiver operating characteristic (ROC) curves for discriminating patients with stage III/IV from healthy controls had areas under the curves (AUC) of 0.84 and 0.886, respectively. Moreover, ucfDNA integrity LINE1‐266/97 was significantly higher in patients with stage III/IV than in stage I/II and in healthy controls. The AUC of ROC curve for discriminating patients with stage III/IV from healthy controls was 0.800. Furthermore, LINE1‐266 fragment concentration was significantly higher in lymph node metastasis (LNM)‐positive patients relative to LNM‐negative patients. The ROC curve for discriminating LNM‐positive from LNM‐negative patients had an AUC of 0.822.

**Conclusion:**

UcfDNA could serve as a promising biomarker for early detection of NSCLC.

## 1 INTRODUCTION

Cancer remains a leading cause of death worldwide and a serious global public health threat. It is estimated that in 2018, there will be 18.1 million new cases and 9.6 million cancer‐related deaths.^1^ Furthermore, the most commonly diagnosed cancer is lung cancer, which is the leading cause of cancer associated deaths.^1^ Non‐small‐cell lung cancer (NSCLC) is the most common pathological type of lung cancer, accounting for approximately 85% of all lung cancers.^2^ Currently, early lung cancer detection in China is very low, with a 5‐year survival rate of only ~15.6%.^3^ The early stages of lung cancer tend to be asymptomatic, thus resulting in about 75% of patients being at an advanced stage at the time of diagnosis. Current diagnostic methods include chest radiograph, computed tomography (CT) scans, bronchoscopy, and biopsy.^4^, ^5^, ^6^, ^7^ However, these traditional diagnostic methods have many weaknesses, including low sensitivity, specificity, and precision. Therefore, new diagnostic methods and treatment options that are biomarker centric are desirable.

Recently, blood‐derived circulating cell‐free DNAs (cfDNAs) offer a promising pool of candidate biomarkers and have been shown to be relevant when establishing diagnosis or prognosis for various malignancies.^8^, ^9^, ^10^, ^11^, ^12^ Additionally, an elevated cfDNA concentration has been associated with breast cancer,^13^ lung cancer,^14^ colorectal cancer,^15^ melanoma,^16^ gastric cancer,^17^ and testicular germ cell cancer.^18^ Moreover, cfDNA integrity, calculated as the ratio of long to short DNA fragments, was also higher in patients with colorectal cancer, periampullary cancer, lung cancer, and breast cancer relative to healthy individuals.^13^, ^15^, ^19^, ^20^, ^21^ Studies have shown that DNA released from necrotic malignant tumor cells vary in size, whereas DNA released from apoptotic cells is usually uniformly truncated into 185‐200 bp fragments^22^; thus, longer cfDNA are emerging tumor biomarkers for malignancy detection.^23^

Another promising biomarkers source for detecting malignancies is urine. Urine cell‐free DNA (ucfDNA) is more easily accessible, and ucfDNA‐based diagnostic methods are really noninvasive compared with cfDNA in blood. In addition, several studies have demonstrated that ucfDNA can serve as an important liquid biopsy component for diagnosing urological and non‐urological tumors, as it carries DNA from urinary tract exfoliated cells or from circulation.^24^, ^25^ Until now, the study of ucfDNA in malignancies has mainly involved in gene mutation (*kras* and *braf*) and DNA methylation,^26^, ^27^, ^28^, ^29^ and few studies have examined the potential clinical relevance of ucfDNA concentration and its integrity.

To investigate the potential clinical role of ucfDNA concentration and its integrity in diagnosing NSCLC, quantitative real‐time PCR (qPCR), targeting long interspersed nuclear element 1 (LINE1), was employed, with two different fragments sizes (97 and 266 bp) examined. Herein, ucfDNA concentration and its integrity were evaluated in 55 NSCLC patients and 35 healthy controls. This study focused on LINE1 since it is one of the most abundant sequences in the human genome, comprising approximately 17% of the human genome and with about 520 000 copies per genome.^30^ It was hoped that qPCR of LINE1 repeats could dramatically increase sensitivity and accuracy of detection. In this study, LINE1 fragments concentrations and its integrity were significantly higher in NSCLC patients relative to the healthy controls, suggesting that quantification of LINE1 fragments may serve as a relevant diagnostic biomarker. Furthermore, LINE1‐266 fragment concentration was significantly higher in lymph node metastasis (LNM)‐positive patients than LNM‐negative patients, indicating that assessing ucfDNA concentration could preoperative prediction of LNM in NSCLC patients. In summary, these preliminary analyses highlight the important properties of ucfDNA concentration and its integrity index and provide a new approach for early detection of NSCLC.

## 2 MATERIALS AND METHODS

### 2.1 Clinicopathologic information

Urine samples from 35 healthy individuals and 55 NSCLC patients, including stage I (n = 10), stage II (n = 10), stage III (n = 12), and stage IV (n = 23) were collected between 2017 and 2019 at the Southwest Hospital, Army Medical University. All subjects in this study provided written informed consent, and the study was approved by the Medical Ethics Committee of Southwest Hospital and was conducted in accordance with relevant guidelines and regulations.

### 2.2 Urine samples processing and ucfDNA extraction

Morning urine specimens (80 mL) were collected and centrifuged at 2000 *g* for 10 minutes. Then, the obtained supernatant urine samples were concentrated to 4 mL using a Vivacell 100 centrifugal filter devices (Sartorius). Then, 4 mL concentrated urine samples were centrifuged at 20 000 *g* for 15 minutes. The supernatants were transferred into cryovials and immediately stored at −80°C until further use. Then, ucfDNA was extracted and purified using a QIAamp circulating nucleic acid kit (Qiagen) according to the manufacturer's instructions. The obtained ucfDNA was then quantified using a Qubit^®^2.0 fluorometer (Life Technologies), according to the manufacturer's instructions. The ucfDNA samples were stored at −20°C until further use.

### 2.3 Quantification of LINE1 repeats via qPCR

A consensus human LINE1 (Gene ID: 54596) sequence was targeted for the qPCR reactions. Primers for short and long LINE1 fragments (97 and 266 bp) were taken from literature.^31^, ^32^, ^33^ The reaction mixtures contained 10 μL FastStart Essential DNA Green Master (Roche), 2 μL each forward and reverse primer pair (0.5 μmol/L), 6 μL RNase‐free water, and 2 μL extracted DNA in a total of 20 μL volume. The qPCR reactions were performed in a CFX96 Real‐Time PCR Detection System (Bio‐Rad) under the following conditions: an initial heating step at 95°C for 10 minutes to activate the DNA polymerase, followed 40 cycles of denaturation at 95°C for 10 seconds and annealing at 60°C for 30 seconds. A negative control (no template) was run in each reaction plate. A standard curve (10 ng‐0.1 pg) was generated by preparing serial dilutions of genomic DNA from peripheral blood leukocytes from the healthy controls. The concentration of LINE1 fragments in each sample was quantified using the standard curve and the absolute quantification method according to the CFX96 Real‐Time PCR software instructions (Bio‐Rad). Reactions were performed in triplicate and mean values were calculated.

### 2.4 Measurement of ucfDNA integrity

Concentrations of ucfDNA were determined by measuring the abundances of short and long LINE1 fragments (LINE1‐97, 266 bp). DNA integrity was calculated as the ratio of longer to shorter fragments (LINE1‐266/LINE‐97). Because the annealing sites of LINE1/97 are within the LINE1/266 annealing sites, DNA integrity value would be 1.0 when template DNA is not truncated and 0 when all template DNA is truncated into fragments smaller than 266 bp. The short fragment was regarded as representing the overall ucfDNA concentration.

### 2.5 Statistical analysis

The Mann‐Whitney *U* test was used to compare LINE1 fragments concentration and integrity values between the NSCLC patients and healthy control groups. Mean values for healthy controls and NSCLC patients within each stage were then compared using Dunnett's multiple comparison test. Receiver operating characteristic (ROC) curve and the area under the curve (AUC) was used to assess the diagnostic value in discriminating NSCLC patients from health controls. All statistical analyses were carried out using the SPSS software, and the figures are generated using the GraphPad Prism software. Results are presented as a mean ± standard deviation (SD) and are considered statistically significant if *P* < .05 (two‐tailed).

## 3 RESULTS

### 3.1 Clinical and pathologic characteristics of NSCLC patients

The study examined 55 patients with NSCLC, including 31 males and 24 females, as well as 35 healthy controls. For NSCLC patients, the mean age was 55 ± 12 years, and for the healthy controls, it was 45 ± 10 years. There was no statistical difference between groups regarding gender or age. Clinicopathologic characteristics of NSCLC patients are presented in Table 1, with NSCLC patients classified into stages I, stage II, stage III, and stage IV based on the tumor node metastasis (TNM) staging system.

**TABLE 1:** Clinicopathologic characteristics of NSCLC patients

Variable	Patients (n = 55)	
	No.	%
Sex		
Male	31	56.36
Female	24	43.64
UICC primary tumor		
T1	15	27.27
T2	8	14.55
T3	16	29.09
T4	16	29.09
UICC regional lymph nodes		
N0	17	30.92
N1	9	16.36
N2	3	5.45
N3	26	47.27
UICC distant metastasis		
M0	32	58.18
M1	23	41.82
UICC stage		
I	10	18.18
II	10	18.18
III	12	21.82
IV	23	41.82

Abbreviations: NSCLC, non‐small‐cell lung cancer; UICC, Union for International Cancer Control.

### 3.2 Concentration and ROC analysis of LINE1 fragments in NSCLC patients

Urine samples were collected preoperatively and ucfDNA (LINE1‐97, 266 bp) concentration and integrity were assessed. The mean LINE1‐97 fragment concentrations in healthy controls and NSCLC patients with stage I/II and stage III/IV were 603.69, 747.59, and 1384.79 pg/mL, respectively. The mean LINE1‐97 value was significantly higher in patients with stage III/IV than in stage I/II and in healthy controls (*P* = .005 and *P* = .003, respectively; Figure 1). A trend of elevation in stage I/II was observed, but the difference of LINE1‐97 value between healthy controls and patients with stage I/II was not significant (*P* = .515). To assess the ability of LINE1‐97 to distinguish NSCLC patients from healthy controls, ROC curve were generated and the AUC values for the stage I/II and stage III/IV groups were 0.627 (0.476‐0.779) and 0.840 (0.747‐0.933), respectively (Table 2). In the detection of NSCLC patients with stage I/II, sensitivity was 0.60, and specificity was 0.71 (Table 2).

**FIGURE 1:** Concentration of LINE1‐97 fragment in healthy controls and NSCLC patients. (A) The mean concentration of LINE1‐97 fragment in patients with stage III/IV was significant higher than in stage I/II and in healthy controls. (B) ROC curve with AUC values for discriminating NSCLC patients from healthy controls

**TABLE 2:** Diagnostic ability of LINE1 fragments in NSCLC patients

	Cut‐off (pg/mL)	Sensitivity	Specificity	AUC (95% CI)
LINE1‐97				
Stage I/II	744.70	0.60	0.71	0.627 (0.476‐0.779)
Stage III/IV	835.70	0.60	0.71	0.840 (0.747‐0.933)
Stage I/IV	668.3	0.89	0.60	0.763 (0.662‐0.863)
LINE1‐266				
Stage I/II	29.64	0.80	0.70	0.551 (0.395‐0.707)
Stage III/IV	148.9	0.60	0.71	0.886 (0.809‐0.962)
Stage I/IV	134.40	0.73	0.71	0.764 (0.665‐0.863)
LINE1‐266/97				
Stage I/II	0.07	0.50	0.80	0.594 (0.435‐0.753)
Stage III/IV	0.17	0.60	0.89	0.800 (0.696‐0.904)
Stage I/IV	0.12	0.62	0.60	0.657 (0.544‐0.770)

Abbreviations: AUC, area under the curve; CI, confidence interval; LINE1, long interspersed nuclear element 1; NSCLC, non‐small‐cell lung cancer.

Similarly, the mean LINE1‐266 fragment concentrations in healthy controls and patients with stage I/II and stage III/IV were 65.20, 72.52, and 245.11 pg/mL, respectively. The mean LINE1‐266 value was also significantly higher in patients with stage III/IV than in stage I/II and in healthy controls (*P* = .0014 and *P* = .0012, respectively; Figure 2). However, there was no significant difference between patients with stage I/II and healthy controls (*P* = .533). Furthermore, the AUC values for discriminating patients with stage I/II and stage III/IV from healthy controls were 0.551 (0.395‐0.707) and 0.886 (0.809‐0.962) (Table 2). In addition, in the detection of NSCLC patients with stage I/II, sensitivity was 0.80, and specificity was 0.70 (Table 2). These results suggested that quantification of LINE1 fragments of various sizes could be used to differentiate NSCLC patients from healthy controls.

**FIGURE 2:** Concentration of LINE1‐266 fragment in healthy controls and NSCLC patients. (A) The mean concentration of LINE1‐266 fragment in patients with stage III/IV was significant higher than in stage I/II and in healthy controls. (B) ROC curve with AUC values for discriminating NSCLC patients from healthy controls

### 3.3 UcfDNA integrity in NSCLC patients and healthy controls

The ucfDNA integrity was calculated as the ratio of LINE1‐266/97. The mean integrity LINE1‐266/97 values in healthy controls and patients with stage I/II and III/IV were 0.108, 0.097, and 0.177, respectively. The mean integrity LINE1‐266/97 value was significantly higher in patients with stage III/IV than in stage I/II and in healthy controls (*P* = .021 and *P* = .035, respectively; Figure 3). However, there was no significant difference between patients with stage I/II and healthy controls (*P* = .778). Furthermore, the AUC values for discriminating patients with stage I/II and stage III/IV from healthy controls were 0.594 (0.435‐0.753) and 0.800 (0.696‐0.904) (Table 2). These findings indicated that ucfDNA integrity LINE1‐266/97 could be used to discriminate NSCLC patients from healthy controls.

**FIGURE 3:** Evaluation of ucfDNA integrity LINE1‐266/97 in healthy and NSCLC patients. The mean ucfDNA integrity LINE1‐266/97 in patients with stage III/IV was significantly higher than in stage I/II and in healthy controls. (B) ROC curve for discriminating NSCLC patients from healthy controls

### 3.4 Correlation between LINE1 fragments concentration and lymph node metastasis

Lymph node metastasis is one of the main means of transfer in lung cancer, and it is also an important factor for the staging and prognosis of lung cancer; thus, we compared the concentration of LINE1 fragments in LNM‐positive patients and LNM‐negative patients. The concentration of LINE1‐97 fragment in 17 LNM‐negative patients and 38 LNM‐positive patients was 876.35 and 1276.88 pg/mL; the concentration of LINE1‐266 fragment in 17 LNM‐negative patients and 38 LNM‐positive patients was 77.27 and 209.75 pg/mL, respectively. The concentration of LINE1‐266 fragment was significantly higher in LNM‐positive patients than LNM‐negative patients (*P* = .009, Figure 4). However, the difference of LINE1‐97 fragment concentration between LNM‐positive patients and LNM‐negative patients was not significant (*P* = .059, Figure 4). Furthermore, the AUC of ROC curve for discriminating LNM‐positive patients from LNM‐negative patients by LINE1‐266 fragment was 0.822 (95% CI: 0.682‐0.962). These results suggested that quantification of LINE1‐266 fragment could be used to predict LNM in NSCLC patients.

**FIGURE 4:** Correlation between LINE1 fragments concentration and LNM. (A, B) Comparing concentration of LINE1 fragments in LNM‐positive and LNM‐negative patients. The concentration of LINE1‐266 fragment in LNM‐positive patients was significantly higher than in LNM‐negative patients. (C, D) ROC curves for discriminating LNM‐positive patients from LNM‐negative patients based on LINE1‐97 or LINE1‐266 fragment concentration

## 4 DISCUSSION

Urine represents an important and promising noninvasive source of biomarkers for diagnosing malignancies. Compared with blood, cfDNA isolation from urine is technically simpler, due to urine containing fewer interfering proteins.^34^ Furthermore, ucfDNA serve an important liquid biopsy component that can enable the detection of both urological and non‐urological tumors, as it carries DNA information from circulation or urinary tract exfoliated cells.^24^ Recently, the studies of ucfDNA have predominantly focused on gene mutation^26^, ^27^ and/or DNA methylation^28^, ^29^; few studies have evaluated ucfDNA concentration or its integrity as a potential diagnostic biomarker.

The aim of this study was to assess the potential application of ucfDNA (LINE1‐97, 266 bp) concentration and/or its integrity as biomarker for early diagnosis of NSCLC. To achieve this objective, LINE1 concentration and integrity were determined by using qPCR. Why did we choose LINE1 as the target of detection? The different sequence targets such as the *β‐actin* gene, and *Leptin*, and amyloid beta precursor protein gene *APP* have been used for the real‐time PCR‐based diagnosis of several types of malignancies, but LINE1, which was used in our study, because of it is one of the most abundant sequences in the human genome, comprising approximately 17% of the human genome and with about 520 000 copies per genome, which are believed to increase the sensitivity of detection of low abundance cfDNA.^30^

Previous studies have demonstrated that an elevated cfDNA concentration can be associated with various types of cancers^13^, ^14^, ^15^, ^16^, ^17^, ^18^; in this present study, ucfDNA concentrations (LINE1‐97, 266 bp) in NSCLC patients were significantly higher than in healthy controls, which is consistent with the findings of previous studies done in blood. Furthermore, ROC analysis indicated that LINE1‐97 fragment had higher sensitivity in distinguishing NSCLC patients from healthy controls; LINE1‐226 fragment had higher specificity in differentiating NSCLC patients from healthy controls. These results suggested that combine fragment LINE1‐97 and LINE1‐226 could increase sensitivity and specificity of detection NSCLC patients. When examining demographic characteristics (age and gender) between NSCLC patients and healthy controls groups, no statistical difference was noted, which is consistent with previous findings in a plasma‐based study.^35^ Furthermore, ucfDNA integrity was significantly higher in patients with stage III/IV than in healthy controls, which is consistent with the previous studies.^13^, ^15^, ^19^ However, we consider ucfDNA integrity was not a significant diagnosis indicator in detection of NSCLC patients based on lower AUC value (AUC = 0.657, 95% CI: 0.544‐0.770). One possible reason that the integrity was not a significant indicator may be due to the type of sequence and/or fragment length of the targeted element compared to other studies.^17^, ^36^, ^37^, ^38^ Another possibility is that ucfDNA degrade more easily than cfDNA in the blood.^39^ It is also possible that ucfDNA is innately shorter than blood‐derived cfDNAs, thus resulting in the target being undetected. What's more, the AUC values for LINE1 fragments concentration were significantly higher than ucfDNA integrity, indicating that quantification of LINE1 fragments concentration is more informative than ucfDNA integrity when attempting to detect NSCLC patients.

In addition to ucfDNA concentration being useful for identifying NSCLC patients, an elevated ucfDNA concentration was also found to be significantly correlated with LNM‐positive patients relative to LNM‐negative patients. Besides, the ucfDNA integrity value was also significantly higher in LNM‐positive patients than in LNM‐negative patients. The AUC of the ROC for discriminating LNM‐positive patients from LNM‐negative patients by ucfDNA integrity was 0.899 (95% CI: 0.816‐0.983). These findings suggested that quantification of ucfDNA concentration could preoperative prediction of LNM in NSCLC patients.

In conclusion, this preliminary study showed that LINE1 fragments concentration and its integrity were significant higher in NSCLC patients with stage III/IV than in healthy controls, which might be a promising biomarker for early detection of NSCLC.

## ETHICAL APPROVAL

The research project was approved by the ethics committee of Southwest Hospital, Army Medical University (Chongqing, China). We have consensus with all participants. All the procedures were done under the Declaration of Helsinki and relevant policies in China.
